The article "Impact of a family history of cardiovascular disease on prevalence, awareness, treatment, control of dyslipidemia, and healthy behaviors: Findings from the Korea National Health and Nutrition Examination Survey" was published in 2021. Journal: PLoS One.

# Impact of a family history of cardiovascular disease on prevalence, awareness, treatment, control of dyslipidemia, and healthy behaviors: Findings from the Korea National Health and Nutrition Examination Survey

**DOI:** 10.1371/journal.pone.0254907

**Published:** 2021-07-29

**Authors:** Seung Jae Kim, Oh Deog Kwon, Eung-Joon Lee, Sun Myeong Ock, Kyung-Soo Kim

**Affiliations:** 1 Department of Family Medicine, Seoul St. Mary’s Hospital, College of Medicine, The Catholic University of Korea, Seoul, Republic of Korea; 2 International Healthcare Center, Seoul St. Mary’s Hospital, College of Medicine, The Catholic University of Korea, Seoul, Republic of Korea; 3 Movinci Clinic, Seoul, Republic of Korea; 4 Department of Neurology, Seoul National University Hospital, Seoul, Republic of Korea; 5 Department of Family Medicine, Yeouido St. Mary’s Hospital, College of Medicine, The Catholic University of Korea, Seoul, Republic of Korea; Federation University Australia, AUSTRALIA

## Abstract

**Background:**

Family history (FH) is one of important risk factors for cardiovascular disease (CVD). However, little is known about its impact on dyslipidemia prevalence and management status. Thus, we aimed to investigate the impact of FH of CVD on dyslipidemia prevalence, awareness, treatment, control, and healthy behaviors in Korean adults.

**Methods:**

We conducted a cross-sectional study using representative data from the Korea National Health and Nutrition Examination Survey (KNHANES) 2014–2018. A total of 22,024 participants aged ≥ 19 years without histories of CVDs were classified into two groups according to the presence of FH of CVD (with FH, n = 3,778; without FH, n = 18,246). FH of CVD was defined as having a first-degree relative with ischemic heart disease or stroke. Multivariate logistic regression analyses were performed to evaluate the association between FH of CVD and dyslipidemia prevalence, awareness, treatment, control, and healthy behaviors (weight control, non-smoking, non-risky drinking, sufficient physical activity, and undergoing health screening).

**Results:**

FH of CVD was significantly associated with a higher dyslipidemia prevalence (adjusted odds ratio [aOR] 1.34, 95% confidence interval [CI] 1.18–1.51), better awareness (aOR 1.54, 95%CI 1.19–2.00), and treatment rates (aOR 1.34, 95%CI 1.12–1.60), but not control. Having an FH of CVD was not predictive of any healthy behaviors in dyslipidemia patients. For non-dyslipidemia patients, FH of CVD even showed significant association with smoking (aOR 1.18, 95%CI 1.02–1.36), and risky drinking (aOR 1.20, 95%CI 1.03–1.40) while it was predictive of receiving health screening (aOR 1.14, 95% CI 1.02–1.27).

**Conclusions:**

Having an FH of CVD might positively trigger dyslipidemia patients to start pharmacological intervention, but not non-pharmacological interventions. Therefore, physicians should make more efforts to educate and promote the importance of non-pharmacological behavioral modification in dyslipidemia patients with an FH of CVD.

## Introduction

Globally, cardiovascular disease (CVD) is the leading cause of mortality [1,2] and management of dyslipidemia is an essential factor for the primary prevention of CVD [3,4]. In addition, family history (FH) is known to be an independent risk factor for CVDs, such as ischemic heart disease and stroke [5–8]. Thus, those with an FH of CVD would need extra attention when managing dyslipidemia for the primary prevention of CVD. In fact, various guidelines on the management of dyslipidemia including 2018 American College of Cardiology/American Heart Association (ACC/AHA) guidelines, 2019 European Society of Cardiology/European Atherosclerosis Society (ESC/EAS) guidelines and the Korean Society of Lipid and Atherosclerosis (KSoLA)’s 2018 guideline, the FH of premature coronary heart disease (CHD) is one of the major risk factors of CVD that modify treatment goals in patients with dyslipidemia [9–11]. Furthermore, all three guidelines mentioned above and 2019 ACC/AHA guidelines on the primary prevention of CVD emphasize not only pharmacological therapy for dyslipidemia, but also non-pharmacological behavioral modifications (e.g., weight control, increasing physical activity, smoking cessation, etc.) for the control of dyslipidemia and the primary prevention of CVD [3,9,10]. There have been a number of previous studies conducted in various countries regarding the prevalence, awareness, treatment, and control of dyslipidemia [12–15]. However, studies that investigated the rates of dyslipidemia in patients with an FH of CVD are relatively rare. Furthermore, the results of studies that examined the healthy behaviors of patients with an FH of CVD compared to those without an FH have been inconsistent. Some studies reported that an FH of CVD did not predict healthy behaviors [16–18] whereas other studies did [19,20]. In addition, few studies have analyzed the association between healthy behaviors and FH of CVD among patients with dyslipidemia. Thus, using nationally representative sample data from the Korea National Health and Nutrition Survey (KNHANES), the purpose of this study was to investigate the impact of an FH of CVD on the prevalence, awareness, treatment, control of dyslipidemia, and the practice of healthy behaviors for the primary prevention of CVD.

## Methods

### Study population

KNHANES is a cross-sectional nationwide survey, representing the non-institutionalized civilian population of Korea, that has been conducted on an annual basis since 1998 by the Korea Centers for Disease Control and Prevention (KCDC). The KNHANES is composed of three parts: a health interview survey, health examination, and a nutrition survey. The selection of participants for KNHANES are performed using a complex, multi-stage, and probability sampling to gather unbiased nationally representative data. The details and representativeness of the KHNANES have been discussed in previous studies [21,22]. This study analyzed data from the KNHANES between 2014 and 2018. Among the 39,199 participants from the KNHANES 2014–2018, those who were younger than 19 years (N = 7,889) were excluded in order to include only the adults. Furthermore, to determine the association between an FH of CVD and prevalence, awareness, treatment, and control status of dyslipidemia, and the practice of healthy behaviors for primary prevention of CVD, those with a prior diagnostic history of CVD (N = 1,413) were excluded. Diagnosis of CVD was defined as a self-report of a prior diagnosis of ischemic heart disease (myocardial infarction or angina) or stroke that was confirmed by a doctor. Ineligible participants with missing values for an FH of CVD, outcome variables, and confounders (N = 7,873) were also excluded, leading to a final study population for analysis of 22,024. We then divided the study participants into two groups according to the presence of an FH of CVD. Participants with an FH of CVD were defined as participants who responded positively to the questions from the health interview survey of KNHANES that were probing if any of their first-degree relatives (parents or siblings) were ever diagnosed with ischemic heart disease (myocardial infarction or angina) or stroke. Subsequently, 3,778 participants with and 18,246 without an FH of CVD were included in the final analysis (Fig 1). This study was approved by the institutional review board (IRB) of the Seoul St. Mary’s Hospital, Catholic University of Korea (IRB approval number: KC20ZASI0909). The requirement for written informed consent was waived.

**Fig 1:** Flow chart of selection process of study population. KNHANES, Korea National Health and Nutrition Examination Survey; CVD, cardiovascular disease.

### Definitions of variables

Using the risk stratification suggested by 2018 KSoLA guidelines for the management of dyslipidemia, the prevalence of dyslipidemia was defined as the proportion of participants with low-density lipoprotein cholesterol (LDL-C) higher than each individual’s desirable levels according to their categorized risk groups (LDL-C ≥160 mg/dL for the low risk group, ≥130 mg/dL for the moderate risk group, and ≥100 mg/dL for the high risk group) [10], a previous diagnosis of dyslipidemia by a physician or those who were currently treated with lipid lowering agents. Awareness of dyslipidemia was defined as a positive response to prior diagnosis of dyslipidemia by a physician among those with dyslipidemia. Treatment of dyslipidemia was defined as those taking lipid-lowering agents among participants with dyslipidemia. Control of dyslipidemia was defined as the proportion of participants who achieved LDL-C goals for each risk group among those treated for dyslipidemia. Both the risk stratification and LDL-C goals for the treatment of dyslipidemia for each risk group suggested by 2018 KSoLA guidelines were generally based on the National Cholesterol Education Program-Adult Treatment Panel III [10,23]. The prevalence of hypertension was defined as the proportion of participants with systolic blood pressure ≥140 mmHg or diastolic blood pressure ≥90 mmHg, a previous diagnosis of hypertension by a physician or those who were currently treated with antihypertensive agent. Prevalence of diabetes mellitus (DM) was defined as the proportion of patients with fasting blood glucose (FBS) ≥126 mg/dl or glycated hemoglobin (HbA1c) ≥6.5%, a previous diagnosis of DM by a physician or those who were currently treated with oral hypoglycemic agent (OHA) or insulin. Overweight and obese participants were defined using body mass index (BMI) values according to the Korean obesity standards (23–24.9 kg/m^2^ for overweight and ≥25.0 kg/m^2^ for obese) [24]. Variables regarding healthy behaviors were derived from the results of a health behavior survey, which is a subcategory of the health interview. The overweight and obese participants who responded positively to making efforts to lose weight were considered as the “weight control” group. As for the smoking status, participants were categorized into either “non-smoker” or “current smoker” groups, with the non-smokers consisting of never-smokers and former-smokers. Risky drinkers were defined as those who drank twice or more a week with an average of 7 or more standard drinks per occasion for men or 5 or more standard drinks per occasion for women. Non-drinkers and persons who drink less alcohol than risky drinkers were considered non-risky drinkers. The degree of physical activity was defined based on the Physical Activity Guidelines for Americans, 2^nd^ edition (PAG) [25]. The PAG states that adults are required to have at least 150 minutes of moderate-intensity aerobic physical activity or at least 75 minutes of vigorous-intensity aerobic physical activity per week or its equivalent combination of moderate and vigorous-intensity activity [25]. Thus, participants who fulfilled the criteria were classified into the “sufficient physical activity” group. To evaluate if participants were actively receiving health screening tests regularly for the prevention of CVD, we also examined the proportion of participants who responded positively to a survey question that asked whether they underwent health screening within the last 2 years.

### Anthropometric and laboratory measurements

Each participant underwent blood work during the survey after fasting for at least 8 hours (12 hours for triglyceride (TG)). All obtained blood samples were immediately processed, refrigerated, and delivered in cold storage to the central laboratory. The transported samples were all analyzed within 24 h. Total cholesterol (TC), high-density lipoprotein cholesterol (HDL-C), triglycerides (TG), and FBS were evaluated with a Hitachi Autonomic Analyzer 7600–210 (Hitachi, Japan), while HbA1c was measured using a Tosoh G8 (Tosoh, Japan). The LDL-C level was obtained using the Friedewald formula (LDL-C = TC—HDL-C +TG/5) when the TG level was <200 mg/dL, while it was directly measured when the TG level was ≥200 mg/dL [14,26]. We also calculated the LDL-C using the Friedewald formula for participants with values of TC, TG, and HDL-C, but had missing LDL-C values. Blood pressure (BP) was obtained by applying the standard protocol according to the AHA’s determination of BP by sphygmomanometry [27]. It was measured 3 times on the right arm of the participant in a sitting position using a mercury sphygmomanometer (Baumanometer; WA Baum Co Inc., Coptague, NY, USA) after resting for at least 5 min. The final BP was determined by averaging the second and third BP readings [14].

### Confounders

Confounding variables reflected in the present study were age, sex, marital status, educational status, employment status, household income, residential area, type of health insurance, level of self-rated health, prevalence of hypertension, prevalence of DM, and BMI. The definitions of the prevalence of hypertension and DM and calculation of BMI are mentioned above. Other confounders were derived from the self-administered questionnaire of the health interview survey of KNHANES.

### Statistical analysis

Sampling weights were applied to all statistical analyses, as designated by the KCDC to reflect the entire Korean general population without bias [21,22]. The sampling weights for each sample participant were constructed based on three factors: the inverse of selection probabilities (primary sampling unit; household); an adjustment for nonresponse (household, person); and a post-stratification to make the calculated survey estimates approximately equivalent to the total Korean population [21]. The characteristics and outcome variables of patients with and without an FH of CVD were compared by means and standard deviations or percentages and standard errors. We performed adjusted Wald test for means and chi-square test for proportions to evaluate the statistical differences of the variables between those with and without an FH of CVD. Moreover, multivariate logistic regression analysis was performed to assess the association between the presence of an FH of CVD and prevalence, awareness, treatment, control of dyslipidemia, and healthy behaviors, with adjustments being made for all of the confounding factors mentioned above. For the outcomes regarding healthy behaviors, subgroup analyses were additionally performed, according to the morbidity status of dyslipidemia. F-adjusted mean residual tests were performed to assess goodness of fit for each multivariate logistic regression model. All analyses were conducted using STATA 14.1 (Stata Corp., College Station, TX, USA). P-values <0.05 were regarded as statistically significant.

## Results

### Baseline characteristics

The baseline characteristics of all study participants, those with and without FH of CVD are summarized in Table 1.

**Table 1:** Baseline characteristics of participants according to the family history of cardiovascular disease^a^.

Characteristics	All (n = 22,024) % (SE) or mean±SD	No family history (n = 18,246) % (SE) or mean±SD	Family history (n = 3,778) % (SE) or mean±SD	P value
Socio-demographic factors				
Sex				0.001
Male	49.5 (0.3)	50.0 (0.4)	46.4 (1.0)	
Female	50.5 (0.3)	50.0 (0.4)	53.6 (1.0)	
Age (years)	44.7±17.8	43.6±18.9	50.4±27.2	<0.0001
Marital status				<0.0001
Married	66.3 (0.5)	35.9 (0.6)	21.8 (0.9)	
Single/divorced/separated/widowed	33.7 (0.5)	64.1 (0.6)	78.2 (0.9)	
Educational status				<0.0001
Middle school or lower	17.4 (0.4)	16.7 (0.4)	21.2 (0.8)	
High school	28.0 (0.5)	27.0 (0.5)	33.1 (0.9)	
College or higher	54.6 (0.6)	56.3 (0.7)	45.7 (1.1)	
Employment status				0.238
Manual	22.4 (0.5)	22.2 (0.5)	23.6 (0.9)	
Non-manual	44.3 (0.5)	44.5 (0.5)	43.4 (1.0)	
Others (students or housewives)	33.3 (0.4)	33.3 (0.4)	33.0 (0.9)	
Income				0.267
Low	12.4 (0.4)	12.5 (0.4)	12.0 (0.7)	
Lower middle	23.2 (0.5)	23.1 (0.5)	23.7 (0.9)	
Upper middle	31.2 (0.6)	31.5 (0.6)	30.0 (1.0)	
High	33.1 (0.7)	32.9 (0.7)	34.3 (1.1)	
Residential area				0.565
Urban	64.6 (0.9)	64.7 (1.0)	64.1 (1.2)	
Rural	35.4 (0.9)	35.3 (1.0)	35.9 (1.2)	
Health insurance				0.915
Medicare	97.0 (0.2)	97.0 (0.2)	97.0 (0.4)	
Medical aid	3.0 (0.2)	3.0 (0.2)	3.0 (0.4)	
Health status				
Body mass index (kg/m^2^)	23.8±3.1	23.7±3.4	24.1±6.5	<0.0001
Overweight or obesity	55.7 (0.4)	55.0 (0.5)	59.5 (0.9)	<0.0001
Self-rated health				<0.0001
Very poor/poor	15.3 (0.3)	14.6 (0.3)	19.1 (0.7)	
Fair	52.4 (0.4)	52.2 (0.4)	53.2 (1.0)	
Good/Excellent	32.3 (0.4)	33.2 (0.4)	27.7 (0.9)	
Prevalence of chronic diseases				
Hypertension	22.8 (0.4)	20.1 (0.4)	32.5 (0.9)	<0.0001
Diabetes mellitus	9.0 (0.2)	8.6 (0.2)	11.3 (0.6)	<0.0001
Dyslipidemia	15.5 (0.3)	14.1 (0.3)	23.1 (0.7)	<0.0001
Healthy behaviors				
Weight control^b^	70.8 (0.5)	70.1 (0.5)	70.2 (1.2)	0.585
No smoking	78.2 (0.4)	78.0 (0.4)	79.3 (0.9)	0.162
Non-risky drinking	86.8 (0.3)	86.8 (0.3)	86.3 (0.7)	0.485
Sufficient physical activity	50.1 (0.5)	51.4 (0.5)	48.4 (1.0)	0.003
Health screening within the last 2 years	64.6 (0.4)	63.2 (0.5)	72.1 (0.9)	<0.0001

All data were weighted to the standard Korean population.

^a^At least one first-degree relative with ischemic heart disease or stroke.

^b^The analysis included only those who are overweight or obese (n = 12,373).

P values were obtained by adjusted Wald test for means or chi-square test for proportions.

Abbreviation: SE, standard error; SD, standard deviation.

### Association between FH of CVD and prevalence, awareness, treatment, and control rates of dyslipidemia

The awareness and treatment rates of dyslipidemia were 76.9% and 46.7% respectively. In addition, the control rate among those treated for dyslipidemia was 23.4%. Dyslipidemia patients with an FH of CVD had significantly higher awareness (84.1% vs. 74.7%) and treatment (54.8% vs. 44.2%) rates than those without an FH of CVD. In terms of control of dyslipidemia, the FH of CVD group had significantly lower rate than the non-FH group (19.6% vs 24.8%) (Table 2). The results of the multivariate logistic regression analysis for the prevalence, awareness, treatment, and control of dyslipidemia between those with and without an FH of CVD are also shown in Table 2. The presence of an FH of CVD was significantly associated with an increased risk of dyslipidemia prevalence (adjusted odds ratio [aOR] 1.34, 95% confidence interval [CI] 1.18–1.51), awareness (aOR 1.54, 95% CI 1.19–2.00), and treatment (aOR 1.34, 95% CI 1.12–1.60). However, an FH of CVD was not significantly associated with the control of dyslipidemia. All multivariate logistic regression models showed good fit (F-adjusted mean residual tests, P values: <0.0001).

**Table 2:** Association between family history of cardiovascular disease^a^ and the prevalence, awareness, treatment and control of dyslipidemia.

Variables	All (n = 22,024)	No family history (n = 18,246)	Family history (n = 3,778)	P value
All (n = 22,024)				
Dyslipidemia prevalence				
Proportion [% (SE)]	15.5 (0.3)	14.1 (0.3)	23.1 (0.7)	<0.0001
Adjusted OR^b^ (95% CI)		1 (reference)	1.34 (1.18–1.51)	<0.0001
Participants with dyslipidemia (n = 4,153)				
Awareness				
Proportion [% (SE)]	76.9 (0.8)	74.7 (0.9)	84.1 (1.3)	<0.0001
Adjusted OR^b^ (95% CI)		1 (reference)	1.54 (1.19–2.00)	0.001
Treatment				
Proportion [% (SE)]	46.7 (0.9)	44.2 (1.0)	54.8 (1.8)	<0.0001
Adjusted OR^b^ (95% CI)		1 (reference)	1.34 (1.12–1.60)	0.001
Participants treated for dyslipidemia (n = 2,087)				
Control				
Proportion [% (SE)]	23.4 (1.1)	24.8 (1.3)	19.6 (1.9)	0.030
Adjusted OR^b^ (95% CI)		1 (reference)	0.76 (0.49–1.17)	0.214

All data were weighted to the standard Korean population.

^a^At least one first-degree relative with ischemic heart disease or stroke.

^b^Adjusted for age, sex, marital status, educational status, employment status, income, residential area, type of health insurance, body mass index, level of self-related health, prevalence of hypertension, and prevalence of diabetes mellitus.

P values were obtained by chi-square test for proportions.

Adjusted odds ratios and their corresponding P values were obtained by multivariate logistic regression analyses.

Abbreviation: SE, standard error; OR, odds ratio; CI, confidence interval.

### Association between FH of CVD and healthy behaviors

According to the multivariate analysis for FH of CVD and the healthy behaviors of all the participants, undergoing health screening within the last 2 years (aOR 1.16, 95% CI 1.05–1.28) was significantly associated with the presence of an FH of CVD. However, having an FH of CVD was rather predictive of smoking (aOR 1.14, 95% CI 1.01–1.30) and risky drinking (aOR 1.15, 95% CI 1.00–1.32) while no significant correlation was found between an FH of CVD and other healthy behaviors. This trend was consistently found in the subgroup analysis conducted with participants without dyslipidemia (aOR 1.14, 95% CI 1.02–1.27 for undergoing health screening; aOR 1.18, 95% CI 1.02–1.36 for smoking; and aOR 1.20, 95% CI 1.03–1.40 for risky drinking). In terms of those with dyslipidemia, none of the healthy behaviors significantly correlated with FH of CVD. All multivariate logistic regression models showed good fit (F-adjusted mean residual tests, P values: <0.0001) (Table 3).

**Table 3:** Association between family history of cardiovascular disease^a^ and healthy behaviors according to subgroups of dyslipidemia prevalence.

Variables	No family history (reference)	Family history adjusted OR^b^ (95% CI)	P value
All (n = 22,024)			
Weight control^c^	1 (reference)	1.02 (0.90–1.16)	0.776
Smoking	1 (reference)	1.14 (1.01–1.30)	0.038
Risky drinking	1 (reference)	1.15 (1.00–1.32)	0.046
Sufficient physical activity	1 (reference)	1.04 (0.96–1.13)	0.323
Health screening within the last 2 years	1 (reference)	1.16 (1.05–1.28)	0.003
Participants with dyslipidemia (n = 4153)			
Weight control^d^	1 (reference)	1.13 (0.90–1.41)	0.293
Smoking	1 (reference)	0.92 (0.69–1.21)	0.542
Risky drinking	1 (reference)	0.96 (0.71–1.29)	0.768
Sufficient physical activity	1 (reference)	1.15 (0.96–1.38)	0.118
Health screening within the last 2 years	1 (reference)	1.11 (0.90–1.38)	0.332
Participants without dyslipidemia (n = 17,871)			
Weight control^e^	1 (reference)	0.97 (0.83–1.13)	0.674
Smoking	1 (reference)	1.18 (1.02–1.36)	0.022
Risky drinking	1 (reference)	1.20 (1.03–1.40)	0.018
Sufficient physical activity	1 (reference)	1.01 (0.92–1.11)	0.849
Health screening within the last 2 years	1 (reference)	1.14 (1.02–1.27)	0.021

All data were weighted to the standard Korean population.

^a^At least one first-degree relative with ischemic heart disease or stroke.

^b^Adjusted for age, sex, marital status, education status, employment status, income, residential area, type of health insurance, body mass index, level of self-related health, prevalence of hypertension and prevalence of diabetes mellitus.

^c^The analysis included only those who are overweight or obese (n = 12,373).

^d^The analysis included only those who are overweight or obese (n = 3,005).

^e^The analysis included only those who are overweight or obese (n = 9,368).

Analyses were performed by multivariate logistic regression model.

Abbreviations: OR, odds ratio; CI, confidence interval.

## Discussion

In this nationwide cross-sectional study, individuals with an FH of CVD had a significantly higher prevalence of dyslipidemia compared to those without an FH. This suggests that individuals with an FH of CVD are at a higher risk of developing dyslipidemia. In fact, these results are expected because both the FH of CVD and dyslipidemia are well-known risk factors for CVD occurrence [5,28,29]. The results of previous studies were also consistent with ours, as the FH of CVD group displayed significantly higher dyslipidemia prevalence [12,15,30].

In terms of the management of dyslipidemia, our results revealed that the awareness and treatment rates were also significantly higher in the FH of CVD group than in the non-FH group. Furthermore, a positive FH of CVD was independently associated with a better awareness and treatment for dyslipidemia. This tendency could be explained by the Health Belief Model [31,32] as those who believe they are more vulnerable to developing a certain disease are likely be more alert to their health status and make more efforts to reduce the threat of that disease. Thus, patients with an FH of CVD would have likely recognized that their risk for CVD was higher than those without, which may have led to better awareness and higher treatment rates. However, despite these results, control rate of dyslipidemia was found to be significantly lower in FH of CVD group than the non-FH group and having an FH of CVD was not significantly associated with control of dyslipidemia in the multivariate analysis. This may imply that when patients’ lipid levels worsen and reach a point where they would require medical treatment, patients without an FH of CVD would also become conscious on the better control of their potential disease. In addition, once patients with dyslipidemia start taking lipid-lowering agents, the LDL-C level would decrease to a certain point regardless of a positive FH of CVD, resulting in the impact of FH of CVD being less significant on control rates compared to other rates. There have been very few studies that examined the relationship between an FH of CVD and awareness, treatment, and control rates of dyslipidemia. One Chinese study also reported that the awareness and treatment rates were significantly higher in the patients with an FH of CHD compared to those without an FH, but the difference in the control rates between the two groups was insignificant [15]. Further studies investigating the medication-taking behavior, such as adherence to lipid-lowering medications between the FH of CVD and non-FH groups, would be needed to verify our results that an FH of CVD does not predict better control rates of dyslipidemia.

In terms of healthy behaviors for the prevention of CVD, there have been various studies that investigated the relationship between individuals with a positive FH of CVD and risk-reducing behaviors. Among these, the results were inconsistent as positive [19,20], negative [17,18] and no correlation [16,33] between the two have been reported previously. In addition, Imes et al. performed a systematic review of 23 articles and concluded that an individual’s awareness of a positive FH of CVD was not a sufficient predictor of health-related behavioral changes [34]. This conclusion was mostly consistent with our overall results for all participants as having an FH of CVD was positively associated with only undergoing health check-ups while it was either negatively associated (non-smoking and non-risky drinking) or had no significant correlation (weight control and sufficient physical activity) with other healthy behaviors. This trend was also consistently seen in individuals without dyslipidemia. Thus, given the result that those with an FH of CVD had a higher risk of developing dyslipidemia, it is crucial to encourage them to adopt healthier behaviors.

Regarding the healthy behaviors of patients with dyslipidemia, a positive FH of CVD was not associated with any of healthy behaviors for dyslipidemia patients. Given that a positive FH of CVD predicted better awareness and treatment rates for dyslipidemia patients but did not predict any of risk-reducing behaviors, we can assume that having an FH of CVD might positively trigger dyslipidemia patients to start pharmacological intervention, but not non-pharmacological behavioral change. In addition, considering that healthy behaviors such as weight control and sufficient physical activity are one of the most important non-pharmacological interventions that are recommended to dyslipidemia patients for the control of disease [9,10], lack of association between a positive FH of CVD and these behaviors could be another reason for an FH of CVD not predicting the better control of dyslipidemia despite its positive association with better awareness and treatment rates. Hence, physicians should pay more attention to motivating and educating patients with dyslipidemia with an FH of CVD to engage in healthier lifestyles for better control of dyslipidemia and prevention of CVD.

The strength of this study is that we used nationally representative survey data for the analyses. To the best of our knowledge, our study is the first to evaluate not only the effect of an FH of CVD on the prevalence, awareness, treatment, and control of dyslipidemia, but also healthy behaviors in patients without a history of CVD. Moreover, various confounding variables, including sociodemographic factors and health status, were adjusted in the analyses. Thus, we believe that our findings offer a meaningful perspective for the control of dyslipidemia and primary prevention of CVD in individuals with an FH of CVD.

However, our study also had some limitations that need to be addressed. First, due to the nature of the cross-sectional study, the causal relationship between an FH of CVD and outcome variables could not be guaranteed. Second, since a large portion of data used in this study were based on self-reported questionnaires, reporting bias could not be ruled out. Third, we could not fully reflect the KSoLA standard for risk stratification of each participant and its corresponding LDL-C goals since some of the risk factors were not available in the KNHANES. For instance, KSoLA actually includes an FH of premature CHD (male < 55 years, female < 65 years) as a risk factor [10]; however, we included an FH of CHD in general since there was no information regarding the age of the diagnosed family members. In addition, KSoLA also considers patients with carotid artery disease and abdominal aneurysm as a high-risk group [10] but the participants’ diagnosis status of these two conditions could not be reflected because such information was also unavailable in the KNHANES. Thus, theoretically, the prevalence and control of dyslipidemia could have been partially misestimated, but we believe that this would not affect the overall tendency of our results considering the well-established representativeness of KHNANES data. Lastly, due to the lack of information in KNHANES, we could not reflect other potential factors that could affect the awareness, treatment, control of dyslipidemia, and healthy behaviors, such as the participants’ knowledge of higher risk of CVD for those with an FH of CVD, their attitudes toward dyslipidemia and CVD, and rapport between the healthcare provider.

## Conclusions

In this representative nationwide study, a positive FH of CVD was associated with higher prevalence and better awareness and treatment rates of dyslipidemia, but not control. In addition, having an FH of CVD was not predictive of any of risk-reducing behaviors for dyslipidemia patients. Therefore, physicians should make more efforts to educate and promote the importance of non-pharmacological behavioral modification among patients with dyslipidemia who have an FH of CVD.

## Supporting information

S1 Dataset (XLSX)
